# Object-Based Image Retrieval Using the U-Net-Based Neural Network

This article has been retracted.

**DOI:** 10.1155/2021/4395646

**Published:** 2021-11-10

**Authors:** Sandeep Kumar, Arpit Jain, Ambuj Kumar Agarwal, Shilpa Rani, Anshu Ghimire

**Affiliations:** ^1^Department of CSE, Koneru Lakshmaiah Education Foundation, Vaddeswaram, Vijayawada, Andhra Pradesh, India; ^2^Department of CSE, Teerthanker Mahaveer University, Moradabad, Uttar Pradesh, India; ^3^Chitkara University Institute of Engineering and Technology, Chitkara University, Punjab, India; ^4^Department of IT, Neil Gogte Institute of Technology, Hyderabad, India; ^5^Nepal Engineering College, Kathmandu, Nepal

## Abstract

Day by day, all the research communities have been focusing on digital image retrieval due to more internet and social media uses. In this paper, a U-Net-based neural network is proposed for the segmentation process and Haar DWT and lifting wavelet schemes are used for feature extraction in content-based image retrieval (CBIR). Haar wavelet is preferred as it is easy to understand, very simple to compute, and the fastest. The U-Net-based neural network (CNN) gives more accurate results than the existing methodology because deep learning techniques extract low-level and high-level features from the input image. For the evaluation process, two benchmark datasets are used, and the accuracy of the proposed method is 93.01% and 88.39% on Corel 1K and Corel 5K. U-Net is used for the segmentation purpose, and it reduces the dimension of the feature vector and feature extraction time by 5 seconds compared to the existing methods. According to the performance analysis, the proposed work has proven that U-Net improves image retrieval performance in terms of accuracy, precision, and recall on both the benchmark datasets.

## 1. Introduction

Nowadays, digital image techniques lead to the tremendous usage of the image retrieval process on the internet. The image retrieval system retrieves different images over the internet with different captions and labels under each image stored in the database. An image retrieval system that uses content as a search key for browsing is known as content-based image retrieval (CBIR) [1]. The main goal of the CBIR methodology is to extract meaningful information from images such as color shape and texture for effective retrieval. The research community contributed to CBIR in the direction of image properties, relevance feedback, fuzzy color, and texture histogram [2]. The proposed algorithms, color histogram, based on relevant image retrieval (CHRIR) [3, 4], work with the image's low-level features, such as objects' physical features for image retrieval. However, these visual features might not reveal the proper semantics of the image. These algorithms may not suit and may generate erroneous results when considering content images in a broad database. Therefore, to improve the CBIR system's accuracy, region-based image retrieval methods using image U-Net-based segmentation were introduced [5]:

(i) Haar discrete wavelet transform (H-DWT) is a popular transformation technique that transforms any image from the spatial domain to frequency domain. The wavelet transformation method represents a function as a family of essential functions termed wavelets [2, 6, 7]. Wavelet transform extracts signals at different scales while input passes through the low-pass and high-pass filters. Wavelets are increasingly becoming popular because of their multiresolution capability and suitable energy compaction property. Haar wavelet is used to represent an image by computing the wavelet transform. It involves low-pass filtering as well as high-pass filtering operations simultaneously [8]. At each scale, the image is decomposed into four frequency sub-bands, namely LowLow, LowHigh, HighLow, and HighHigh, where Low stands for low frequency and High stands for high frequency. Haar wavelet's function *X*(*t*) can be described as
  (1) $$\begin{array}{c} X\left(t\right)=\left\{\begin{array}{cc} 1, & 0\leq t\leq 0.5,\\ -1, & 0.5\leq t<1,\\ 0, & \text{otherwise}. \end{array}\right\} \end{array}$$
Its scaling function *χ*(*t*) can be defined as *χ*(t) = $\;\left\{\begin{array}{cc} 1, & 0\leq t<1,\\ 0, & \text{otherwise} \end{array}\right\}$.
(ii) Lifting scheme: it is a well-known approach used for the second generation wavelets [5]. It has much potential in CBIR because of its simple structure, low complexity in computation, convenient construction, etc. It has proved its potential in performing iterative primal lifting and dual lifting [9–11] with multiresolution analysis. Using a lifting scheme, we can build wavelets having more vanishing moments and smoothness, thus enabling them to be more adaptable and nonlinear. The lifting scheme is used for designing wavelets and performing wavelet transformation techniques such as discrete wavelet transform (DWT).

Most of the traditional techniques used machine learning techniques, and these techniques work on the whole image, making it a more time-consuming process. Therefore, this paper proposed a U-Net-based neural network for segmentation purposes and Haar DWT and lifting wavelet schemes were used for feature extraction in content-based image retrieval (CBIR). Haar wavelet is preferred as it is easy to understand, very simple to compute, and the fastest. U-Net-based neural network (CNN) gives more accurate results than the existing methodology because deep learning techniques can extract low-level and high-level features from the input image, which is the novelty of this research. In Section 2, we presented a literature survey. In Section 3, we explained our proposed architecture and methodology.  Section 4 discusses the results of 2 benchmark datasets, and Section 5 represents the conclusion section.

## 2. Literature Work

Digital image retrieval and its applications are vast to study. There are many traditional techniques in image retrieval, but the key issue is that various techniques may have different types of variations, i.e., accuracy, error, and detection rate. Many research communities [1–16] proved that object detection and image retrieval error rate are less, as shown in Table 1.

## 3. Proposed Methodology

In Figure 1, the flowchart describes the proposed methodology in which the image retrieval has to be done. The following steps explain the proposed methodology.

### 3.1. Image Acquisition

An image is taken as input which has to be converted into a grayscale image. The converted image is then sent to the preprocessing step for further process. In the acquisition process, the image with Real-World Data is converted into an array of numerical data. The image must be captured with the appropriate camera and converted into a computerized pattern [22–24].

### 3.2. Preprocessing

Preprocessing is performed to remove distortions and other unwanted features while processing the image and extract the proper portion of the image corresponding to the analysis of image retrieval using different algorithms [25–27] such as boundary detection. Preprocessing involves removing unwanted features, resizing the image, boundary detection, and normalization. The image is processed through different phases in preprocessing, such as resize, boundary detection, and normalization.

### 3.3. Segmentation

There are various traditional methods to normalize the image for segmentation, but the U-Net-based neural network detects the object more efficiently.

The proposed methodology used 3-layer U-Net architecture, and it is one of the fully convolutional neural networks which works with very few training models yet yields compelling segmentation results. U-Net consists of a 3-layer convolution neural network, ReLU functions, and pooling functions, and in each layer, the pooling operations are replaced by the upsampling operators such that the network's output gives an image with increased resolution. U-Net performs the classification on every pixel and generates the output with the same size as the input. The U-Net architecture is symmetric and usually has a U shape. The left side of the network is a contracting network, and the right is expanding network. The architecture is shown in Figure 2. Downsampling will be done on the left side of the U-Net architecture, and on the right side, upsampling will be done. Each block in the architecture takes an input and passes through 2 convolution layers, 3 × 3 with a stride of 2 and 2 × 2 max-pooling with the corresponding cropped feature map.  Table 2 shows the full description of the input image with 3 phases of downsampling and upsampling. Once the image is segmented accurately and features can be extracted, the encoding path, i.e., downsampling, is passed through 3 × 3 × 3 convolutions. It is followed by ReLU (rectified linear unit) operation with 16 channels and 2 × 2 × 2 max-pooling with stride 2. It consists of 3 phases/layers of convolution. At each layer, the feature channels get doubled. In total, 11 convolution layers were taken.

### 3.4. Feature Extraction

In this process, the image is reduced using classification to more manageable parts stored as a dataset for further image processing [2, 28–31]. The process is as shown in Figure 3. These large data sets contain many variables that must be processed and need many computing resources to process.

The method of feature extraction used may alter depending upon the traditional and nontraditional methods [32–35]. After segmentation, the YUV component of the input image is extracted as shown in Figure 4. Once the YUV component was extracted, the Sobel and Canny edge detection and wavelet transformation were applied for in-depth feature extraction [36–40]. The entire sequence of feature extraction is shown in Figure 3.

### 3.5. Classification

The extracted data will be in binary format, stored in the database during the enrollment process, or verified with the existing data during the matching process [41–47]. If the similarity index of the image is more, then a similar kind of image will be retrieved. The similarity distance is estimated by Manhattan distance, Euclidean distance and Chebyshev rule. The mathematical formulations are shown as follows:

(2) $$\begin{array}{c} D_{M}=\left|x1-x2\right|+\left|y1-y2\right|,\\ D_{E}=\sqrt{{\left(x1-x2\right)}^{2}+{\left(y1-y2\right)}^{2}},\\ D_{Cheb}=\max\left(\left|x1-x2\right|,\left|y1-y2\right|\right). \end{array}$$

## 4. Results

Overall, GUI is prepared for the proposed work using the MATLAB 2014a tool by taking input of the image as a query image as shown in Figure 3. The entire work was performed on a laptop with the configuration of Intel I3, of NVIDIA graphics card with 4 GB RAM. Various hyperparameters are used in the architecture. A total of 50 epochs is used while training the model. The validation split is considered as 0.1. It considers 90% of the images for the training purpose and 10% for the testing purpose. The dropout value is 0.2; it means that of five inputs, one is excluded from each cycle. Sixteen filters are used for the convolution purpose, and the learning rate lies between 0 and 1. For evaluation of the proposed work, the Corel 1K database and Corel 5K database cover many semantic categories, as shown in Figures 5 and 6. These datasets are widely used for content-based image retrieval techniques. Totally 10800 images are available in the Corel 1K dataset, and they are divided into 80 different groups according to the various categories. The database includes butterflies, horses, bushes, flowers, etc., and each category contains more than 100 images. The users determine the partitioning of the database into meaningful featured categories because of image similarity.

Figure 7 shows the overall GUI of the proposed work. The proposed work gives high accuracy, precision, and recall up to 93.1%, 99.77%, and 87.23%, and 88.39%, 84.75%, and 81.01%, respectively, for Corel 1K and Corel 5K datasets, as shown in Table 3 as well as Figures 8–10. Based on the novel proposed work, feature extraction time reached 4.187 sec, as shown in Table 4 and Figure 11. In Corel 1K benchmark datasets, nine samples were considered for evaluation and similarity matrices of these datasets are shown in Table 5 and Figure 12. In Corel 5K benchmark datasets, 21 various samples were considered for evaluation and similarity matrices of these datasets are shown in Table 6 and Figure 13. The overall precision values of the proposed work are high compared with the existing methodology, and the results are shown in Table 7 and Figure 14. The mathematical formulation of the parameters is shown as follows:

(3) $$\begin{array}{c} \text{accuracy}=100*\left(\frac{\left(\text{TP}+\text{TN}\right)}{N}\right),\\ \text{recall}=\frac{\text{TP}}{\left(\text{TP}+\text{FP}\right)},\\ \text{precision}=\frac{\text{TP}}{\left(\text{TP}+\text{FN}\right)}, \end{array}$$

where TP is true positive, TN is true negative, FN is false negative, FP is false positive, and *N* is the size of the dataset.

## 5. Conclusion

The U-Net-based architecture makes the proposed work different from the existing methods, giving a high detection rate. The U-Net-based neural network detects the object more efficiently. It is a fully convolutional neural network (CNN) that works with very few training models yet yields compelling segmentation results. It is a three-layered segmentation architecture that improves the overall accuracy of our content-based image retrieval system by around 93%. For evaluation of the proposed work, the Corel 1K database and Corel 5K database are used. The results show that accuracy and precision are very high compared to the existing methodology. The feature extraction time of our proposed methodology is also significantly less compared to the MTSD method. Hence, we can conclude that our proposed methodology is very fast, accurate, efficient, and precise compared to the MTSD method.

## Figures and Tables

**Figure 1:** Flow chart of the proposed system.

**Figure 2:** U-Net-based architecture diagram.

**Figure 3:** Flow chart of feature extraction technique.

**Figure 4:** YUV component of the input image.

**Figure 5:** Sample format of the Corel 1K/Wang database (people, beach, buildings, buses, dinosaurs, elephants, flowers, horses, and mountains).

**Figure 6:** Sample format of the Corel 5K database (butterfly, bear, sunset, card, symbol, tiger, sippy, people, vegetable, cloud, beers, trees, doors, cars, bridges, waterfalls, bullock cart, revolver, pattern, flag, and art).

**Figure 7:** GUI of the proposed work.

**Figure 8:** Accuracy comparison of the proposed work with the existing methodology.

**Figure 9:** Precision comparison of the proposed work with the existing methodology.

**Figure 10:** Recall comparison of the proposed work with the existing methodology.

**Figure 11:** Dimension and time comparison of the proposed work with the existing methodology.

**Figure 12:** Similarity metrics on the Corel 1K dataset.

**Figure 13:** Similarity metrics on the Corel 5K dataset.

**Figure 14:** Precision comparison of the proposed work with the existing methodology.

**Table 1:** Comparison of the existing image retrieval techniques.

S. no.	Author	Year	Method/methodology	Comments
1	Liying and Lirong [13]	2017	Scale-invariant feature transform (SIFT)	Performs retrieval on more than a single query to increase the retrieval accuracy.
			Convolutional neural network (CNN)	

2	Dhotre et al. [4]	2017	The color feature extracted through CHRIR and wavelet transform performed using multilevel Haar wavelet transform (MHWT)	Proved to be a faster retrieval method on an image database with one of the physical features. Works more accurately with increased retrieval speed and minimized time.

3	Jayanthi and Karthikeyan [2]	2015	FCTH, CEDD, HWT, and DWT using fuzzy linking and Gabor filters	Database with 1000 color images results in better recall and average precision of retrieval.

4	Thepade and Shinde [3]	2015	Haar wavelet transforms with Canny edge detection based on shape features using gradient techniques such as Prewitt, Laplace, and Sobel, and the slope magnitude technique with the Manhattan similarity function	Database with 350 color images
				Frei-Chen and Sobel give better performance than the other algorithms that used Canny implementation.

5	Jayanthi and Karthikeyan [2]	2015	HWT and DWT using Gabor filters and fuzzy linking	Gives good results in average precision and recall value.

6	Gupta and Kushwah [8]	2015	Haar discrete wavelet transform (H-DWT), gray level co-occurrence matrix (GLCM)	Improved results in comparison with previous methods.
			Support vector machine (SVM)	

7	Agarwal et al. [5]	2014	Used color edge detection and DWT	Database used was Wang's image database. Gave high precision and recall values.

8	Agarwal et al. [5]	2014	Color edge detection, DWT	High precision and recall indicate an exemplary retrieval system
			Canny edge detection	

9	Ying Chen and Wu [6]	2011	Uses optical flow to extract the information from the video; extraction process with Haar wavelet	Locates the feature almost near the query point using index values.

10	Chatzichristofis et al. [7]	2010	The method based on color and edge directivity descriptor (CEDD)	Demonstrated successful retrieval on benchmark datasets.
			Utilizes the binary Haar wavelet transform for extraction	

11	Quellec et al. [12]	2010	The multidimensional wavelet filter bank	Can be used in a different dimension of signal and different lattices.

12	Verma et al. [1]	2009	Texture analysis-based scheme	Own dataset with 100 color images of size 256 × 256 pixels each. Accuracy up to 73%.
			I level Haar wavelet used for image decomposition F-norm theory to decrease the dimension of the extracted feature; fuzzy logic similarity measure used	

13	Huang et al. [10]	2005	Lifting scheme F-norm theory	Good at retrieval.

14	Wong et al. [9]	2005	AdaBoost-based face defection method and the lifting wavelet transform (LFWT) technique	Efficient with small memory to detect the face. Suits best for multimedia applications

15	Munjal and Bhatia [17]	2019	UCID dataset used, CEDD and Gabor wavelet transform (GWT) for feature vector	Accuracy = 91.9%.

16	Varish et al. [18]	2020	Fusion of histograms of gradients and invariant moments, Corel 1K and GHIM-10K dataset used for validation	Precision = 89% and 90%.
				Recall = 17.80% and 3.60.
				F-score = 29.49% and 6.92%.

17	Wadhera and Agarwal [19]	2020	3D center symmetric LBP + Gaussian filter + gray level co-occurrence matrix (GLCM), STex texture, and ESSEX face database	Precision = 61% and 97.4%.
				Retrieval rate = 97.4%.

18	Ajam et al. [20]	2019	LBP + HSV + entropy, Corel 10K and Corel 5K databases used	Retrieval rate = 59.51% and 49.13%.

19	Xiaobo et al. [21]	2021	Adaptive threshold + directional LBP, and Corel 1K database	Precision = 67.63%.

**Table 2:** Complete description of U-Net-based architecture.

Phases	Input image	Convolution layers	Channels	ReLU and max-pooling	Output image	Sampling type	Stride
1	64 × 64 × 40	3 × 3 × 3	16	2 × 2 × 2	32 × 32 × 20	Downsampling	2
2	32 × 32 × 20	3 × 3 × 3	32	2 × 2 × 2	16 × 16 × 10	Downsampling	2
3	16 × 16 × 10	3 × 3 × 3	64	2 × 2 × 2	16 × 16 × 10	Downsampling	2
1	16 × 16 × 10	3 × 3 × 3	32	2 × 2 × 2	32 × 32 × 20	Upsampling	2
2	32 × 32 × 20	3 × 3 × 3	64	2 × 2 × 2	64 × 64 × 40	Upsampling	2
3	64 × 64 × 40	1 × 1 × 1	64	2 × 2 × 2	64 × 64 × 1	Desired sample	2

**Table 3:** Average accuracy, precision, and recall of the retrieval image.

Dataset	MTSD accuracy (%)	Proposed accuracy (%)	MTSD precision (%)	Proposed precision (%)	MTSD recall (%)	Proposed recall (%)
Corel 1K	68.49	**93.01**	56.34	**91.77**	—	**87.23**
Corel 5K	53.39	**88.39**	54.48	**84.75**	—	**81.01**

**Table 4:** Dimension (*D*) of the feature vector and feature extraction time.

Methods	Dimension	Feature extraction time (sec)
MTSD	179	9.1615
Proposed	220	4.1815

**Table 5:** Similarity metrics on the Corel 1K dataset.

Group	*L*1	Euclidean	Chebyshev
People	91.05	79.81	91.76
Beach	87.87	89.27	89.60
Buildings	83.89	87.99	88.82
Buses	79.70	79.92	90.36
Dinosaurs	89.18	90.59	90.01
Elephants	89.66	90.77	88.16
Flowers	90.71	80.39	89.12
Horses	89.73	91.72	87.36
Mountain	87.57	90.89	89.81

**Table 6:** Similarity metrics on the Corel 5K dataset.

Group	*L*1	Euclidean	Chebyshev
Butterfly	81.05	79.24	82.29
Bear	82.70	76.98	79.86
Sunset	80.90	75.15	70.18
Card	77.64	79.11	73.56
Symbol	83.57	81.36	79.09
Tiger	81.16	79.11	82.36
Sippy	83.91	80.08	83.01
People	83.63	81.10	81.73
Vegetable	79.51	79.06	80.17
Cloud	84.10	80.25	82.97
Beers	82.19	81.36	83.97
Trees	80.90	78.15	73.00
Doors	78.18	71.02	74.08
Cars	79.26	74.08	74.83
Bridges	76.82	71.59	76.59
Waterfalls	80.45	76.78	81.08
Bullock cart	83.67	79.71	81.11
Revolver	84.01	80.18	83.31
Pattern	79.11	77.01	77.08
Flag	78.08	76.8	73.12
Art	74.19	79.70	70.14

**Table 7:** Average precision comparison of the proposed work with the existing methodology.

Dataset	Precision of [37] (%)	Precision of [38] (%)	Precision of [39] (%)	Precision of [40] (%)	Precision of [41] (%)	Proposed precision (%)
Corel 1K	75.01	82.09	79.9	69.40	76.60	**91.77**
Corel 5K	—	—	62.97	53.90	59.10	**84.75**

## Data Availability

The data used to support the findings of this study are available from the corresponding author upon request.
